# Study on Influencing Factors and Countermeasures of Elderly Nursing Services in the Elderly

This article has been retracted.

**DOI:** 10.1155/2022/4501228

**Published:** 2022-05-16

**Authors:** Shuo Liu, Li Chen, Dandan Li, Qianqian Yang, Fangfang Liu, Yanli Cheng

**Affiliations:** ^1^Rehabilitation Center for the Aged, Beijing Rehab Hospital, Capital Medical University, Shijingshan District, Badachu Xixiazhuang Gongliao Road, Beijingshan 100144, China; ^2^Gannan Healthcare Vocational College, Ganzhou City, Jiangxi Province 341000, China; ^3^Pharmaceutical Engineering, Pharmaceutical Engineering Part, Jiangsu Ocean University, 222005 Lianyungang, Jiangsu, China

## Abstract

**Methods:**

500 inpatients with chronic diseases in a famous tertiary hospital in a city were studied, and the corresponding countermeasures were put forward through the analysis of their needs and influencing factors. Results. The study found that the vast majority of elderly patients have higher requirements for elderly care services, which is related to factors such as family income. Compared with the huge medical demand, there is a large gap in the level of domestic medical and health talents. According to relevant research, the current number of beds in China is 1 : 0.27, but in fact it is 1 : 0.4. Therefore, relevant units should strengthen the health examination of the elderly, provide high-quality medical services, make full use of health resources, and strengthen nursing management, so as to improve the quality of nursing services.

**Conclusion:**

The survey results show that the vast majority of elderly patients have high requirements for their elderly care services, which is related to family income and other related factors. Therefore, relevant departments should formulate corresponding measures to improve the quality of life of the elderly.

## 1. Introduction

In recent years, with the social awareness of mental health and medical methods changes, more and more people began to pay attention to the mental health of the elderly. Relevant data show that in the elderly patients with chronic diseases, the active use of nursing services can promote their preparation and psychological support and then can effectively reduce the melancholy mood of patients. In the modern medical service mode, nursing, as a more way of care, more reflects the personal feelings of patients and the humanization and professionalism of patients, so it has been generally recognized by medical workers and patients.

According to relevant information, there are about 400 elderly people with chronic diseases or lost self-reliance, with varying degrees of care needs. The service of nursing work not only plays an important role in the elderly patients' disease diagnosis, chronic rehabilitation, end care, and care, but also will continue to their life cycle in their lives.

According to Zhou Yinghong (2020), the establishment of various nursing homes shows that the education level, the number and education level of children, regional environment, and other factors have a significant impact on the demand for life care services of the elderly. In terms of how to improve the effective supply of rural community home-based elderly care services, this paper puts forward community home-based elderly care services that reasonably meet the “good life needs” of rural elderly according to the rural characteristics of each region and the elderly care needs of rural elderly [1]. According to Ma Xiao(2020), with the aggravation of China's aging, by the end of 2015, there will be 222 million people over the age of 60 in China, accounting for more than 16% of the total population. The change of family structure will also bring corresponding pension problems. In this paper, a large number of elderly people are interviewed by questionnaire, and the needs of elderly people for pension services are analyzed by data [2].

With the development of the aging population, some medical institutions have included chronic disease management, rehabilitation care, long-term care, and hospice care into the category of disease care, so as to better meet the people's diversified and multilevel needs of health services. However, in the implementation of nursing services, due to the system is not sound enough, there are still some problems; that is, the quality of nurses is not high, and the management is not standardized. Therefore, this paper aims to investigate the nursing needs of the elderly, and to analyze their relevant factors, in order to continue to improve their countermeasures and plans in the future work [3–8].

This study investigated 500 elderly patients in a well-known class a hospital from April 2018 to April 2019, analyzed the factors affecting the demand for elderly care services, gave corresponding countermeasures, and put forward new research directions for the demand for elderly care services, so as to expand and promote the home care service market for the elderly and to increase the happiness of the elderly in their later years.

## 2. Data and Methods

### 2.1. General Information

From April 2018 to April 2019, a total of 500 elderly patients were selected for the experimental study, including 325 men, 65 to 91 years old, 65 to 91 years old, average age (69.87 ± 15.62), 175 women, 65 to 89 years old, average age (71.69 ± 10.32). There was no significant difference in the overall data (*P* > 0.05).

### 2.2. General Methods

The data were counted into “General Data Survey Form” and “Service Demand Survey Form” for investigation. (1) The general data survey form mainly includes the monthly income, education degree, and self-care ability of the elderly patients.(2) The service demand survey form compiled according to the actual needs of elderly patients and the opinions of relevant departments of the hospital. A total of 500 questionnaires were issued, which were issued and recovered by investigators to ensure the validity of the questionnaire.

### 2.3. Statistical Methods

This section targets the sample of older patients needing care for algorithmic efficacy analysis. Comparative analysis of monthly income, education level and self-care ability. The *R*^2^ values were obtained using a linear regression method under SPSS, and the *t* values and *P* values were obtained using a bivariate *t* calibration.

The *R*^2^ values are counted as the ratio of the regression residue to the mean residue, as shown in

(1) $$\begin{array}{c} R^{2}=\frac{\sum_{i}\left(x_{i}-\bar{x}\right)}{\sum_{i}\left(x_{i}-\tilde{x_{i}}\right)},\overset{¯}{x}=\frac{1}{n}\overset{n}{\underset{i}{\sum }}x_{i}, \end{array}$$

Wherein: the average value calculated by the survey sample sequence; $\tilde{x_{i}}$: The *i*th regression value in the series; *x*_*i*_: The *i*th input value in the sequence; *n*: Number of samples tested.

*T*-value and bivariate *t*-value come from bivariate t-test process, where *t*-value is the value of output result. When *t* > 10.000, the greater the *t*-value, the greater the statistical difference; *P* value is the logarithm of the output result. When *P* < 0.05 and *P* < 0.01, the lower the *p* value, the higher the confidence. According to the length, only the value of *T* (value) is explained here, for example formula

(2) $$\begin{array}{c} t_{\text{Value}}=\frac{\bar{x}-\mu }{\sigma_{x}/\sqrt{n-1}},\bar{x},\mu =\frac{1}{n,m}\overset{n,m}{\underset{i=1}{\sum }}x_{i},\sigma_{x}=\frac{1}{n-1}\sqrt{\overset{n}{\underset{i=1}{\sum }}{\left(x_{i}-\bar{x}\right)}^{2},} \end{array}$$

where it investigates the average value of the sample sequence calculation; 渭: *M* is the average of reference sample sequence; *n* is the number of number of nodes examining the sample sequence; *m* is the number of nodes of the reference sample sequence; and ^*σ*^*x* investigates the standard deviation rate of the sample sequences.

## 3. Results

### 3.1. General Data and General Service Needs Analysis of the Elderly

The analysis of the service needs 500 elderly people, and the results suggest that the general data of education and living ability of 500 elderly patients differ significantly (*P* < 0.05).

In Table 1, culture degree refers to the data samples into junior high school, high school, junior college, or above according to the cultural level. Marriage status refers to dividing the data sample into unmarried and married/widowed two levels according to the marital status. Family income refers to the data sample that is divided into three levels of monthly household income: <3000 yuan, 3000-6000 yuan, and >6000 yuan. Self care ability: the sample data is divided into two types of self-care ability, which cannot be self-care according to self-care ability; Percentage: refers to the data samples divided according to various indicators and their division standards, and the proportion of all samples in the total data samples; Nursing needs: the number of data samples with nursing needs under various classification standards after classification according to various indicators and classification standards; Percentage: divided according to various indicators and division standards. The number of data samples with care needs is a proportion of the total data samples under all kinds of division criteria.

In Figure 1, culture degree refers to the data samples into junior high school, high school, junior college, or above according to the culture level.

In Figure 2, family income refers to the data sample that is divided into three levels: <3000 yuan, 3000-6000 yuan, and >6000 yuan.

In Figure 3, marriage status refers to dividing the data samples into unmarried and married/widowed levels according to the marital status.

In Figure 4, self-care ability refers to the data samples divided into two categories of self-care, one of which if they cannot take care of themselves according to self-care ability.

### 3.2. Logistics Regression Analysis of the Influencing Factors of Nursing Demand

Among the 500 elderly people participating in the study, logistics regression analysis of care impact factors and setting independent variables such as gender, age, education level, and other factors found that self-care ability, education level, and family income were the main factors affecting the needs for examination care (*P* = 0.0001). The remaining independent variables are determined to be meaningless by logistics regression analysis (*P* = 0.0001), as shown in Table 2.

The factors of nursing needs found in Table 2 are as follows: age: data sample age; life nursing: the level of life nursing ability of data samples; education: education and cultural level of data samples; gender: gender index; marital status of the data sample: marriage; household income: the level of household income capacity of the data sample; standard error: describe the discreteness of statistical distribution of corresponding samples and the scale of statistical sampling error of corresponding samples; and degree of freedom: refers to the number of variables when calculating statistics.

At present, retirees aged 65 and over take care of the elderly.

## 4. Problems and Related Geriatric Nursing Countermeasures

The care of the elderly is a long job that runs through their later years. At present, retirees aged 65 and over take care of the elderly. With the development of society and the continuous improvement of medical conditions, various medical institutions are gradually transforming nursing care and according to different conditions, but there are still many problems in practice. At present, professional nurses in health institutions in China generally receive a low education level, and the allocation of medical resources is not perfect. Through the existing medical equipment and medical personnel allocation of a third-class hospital, its needs for elderly patients cannot be met. In view of this, the medical institutions in China should be fully aware of the importance of geriatric nursing work and take corresponding measures to better meet the needs of the elderly.

Elderly care is a long-term work, which runs through their whole old age. At present, most of the people who take care of the elderly are retirees aged 65 and above. Their energy and professional level cannot meet the nursing needs of the existing elderly. With the change of China's population structure and the continuous improvement of medical conditions, medical institutions are gradually transforming nursing according to their own conditions, but there are still many problems in practice. At present, the education level of professional nurses in health institutions in China is generally low, and the allocation of medical resources is still imperfect. Through the medical equipment and medical personnel allocation of the existing tertiary hospitals, their needs for elderly patients cannot be met. In view of this, China's medical institutions should fully understand the importance of elderly care and take corresponding measures to better meet the needs of the elderly.

### 4.1. Major Problems Existing in Geriatric Care

#### 4.1.1. The Gap of Professional Caregivers Is Huge

Compared with the huge medical demand, there is a big gap in the level of domestic medical and health talents. According to the relevant investigation and research, the current number of beds in China is 1 : 0.27, but in reality, it is 1 : 0.4. In addition, in China, the cost of nurses is far lower than the actual medical costs.

#### 4.1.2. Nursing Technology and Level Will Need to Be Improved Urgently

Medical care has the concept of three points of medical treatment and seven points of nursing. At present, based on home care, hospital care is based on home care. Due to the lack of professional and independent medical institutions, there are often repeated and intermittent occupation of beds in secondary and tertiary general hospitals. Due to the cost of long-term care brought about by family care is too high, it is difficult for most families to maintain, and the quality of family care and occupational care is also very different and cannot not fully adapt to clinical needs.

#### 4.1.3. Affected by Nursing Services Institutions

In the process of China's modernization, there are many nursing homes set up for the elderly and community elderly clubs in the society. Especially those community units that specialize in contributing to a variety of benefits for the elderly, they will use various ways to provide the most direct health care to the elderly, giving them more benefits in their lives. These community agencies, while a government policy, can provide various benefits for the elderly for free, are difficult to meet their requirements due to the lack of professional care ideas. Most of the communities provide leisure for the elderly, and have not enough medical resources, which also affects the medical level of the elderly.

#### 4.1.4. Affected by the Family

The problems of the elderly are basically borne by the elderly, and the elderly are also their family and personal problems. With the growth of age, some of their chronic diseases will also have a certain impact on their bodies, but most families do not really cultivate them, especially when their self-protection ability is gradually declining, which is when they need it most. Therefore, the visit, care, and companionship of children are also an important part of the pension. It is the source of happiness and happiness for the elderly and the basic guarantee to improve their quality of survival.

#### 4.1.5. Government Supervision Is Not Enough

In addition, due to the current “medical care,” policy and the lack of management, management, supervision, supervision and management of the elderly, part of the work of elderly care has been left unattended for a long time. Some departments have various contradictions due to unclear responsibilities and non-standard nursing staff, which is very detrimental to the physical and mental health of the elderly.

### 4.2. Countermeasures

#### 4.2.1. Establish a Scientific Nursing Facility

With the acceleration of the population aging process, the old-age care service industry has developed rapidly, and a scientific old-age care service system has also begun to be formed in the developed coastal cities. At the same time, with the support of the government, arranging nursing work for some elderly people with low income and good physical quality can not only bring them economic income, but also meet their needs, which can be said to kill two birds with one stone. In addition, the relevant hospital operation costs are also relatively high, and there will be a large amount of capital investment in the initial stage. The relevant departments should formulate corresponding subsidies and medical security measures to ensure their normal operation.

#### 4.2.2. Provide High-Quality Nursing and Health-Care Services for the Elderly Recognition

At present, in medical institutions, regular physical examination, health consultation, rehabilitation training, and psychological counseling for the elderly are important contents of current elderly care services. However, for the elderly who cannot take care of themselves and have psychological problems, the Chinese health department does not pay enough attention to them. It should not only improve their mental health, but also pay attention to the care and prevention of the elderly, strengthen the care and prevention of the elderly, strengthen the communication with their children, let them offer regular condolences to the elderly, and improve their self-health awareness. Fourth, continue to take care of the elderly who cannot be taken care of and improve the quality of life of the elderly [9–11].

#### 4.2.3. Increase Care Efforts

Once the elderly enter the old age, they will become a vulnerable group. Therefore, more attention is needed. Both the children of the elderly and the staff of communities and nursing homes should strengthen communication and interaction with the elderly, let them feel their warmth and respect, eliminate their loneliness and loneliness, increase their sense of happiness, and let them establish a healthy concept and face life optimistically.

#### 4.2.4. Conduct Regular Health Education

It is very necessary to carry out health knowledge lectures. We should let the elderly understand health knowledge, enhance health awareness, cultivate a good attitude towards life, treat life, have regular physical examination, and improve the quality of life of the elderly.

#### 4.2.5. Establish Good Family Relationships

No matter how good the medical service is, it is not comparable with the warmth of family love. Therefore, we should strengthen the health education and care of the elderly, so that the family and children can better take care of and understand, so as to eliminate the negative psychology of the elderly and let they have a happy old age.

### 4.3. Make Full Use of Existing Health Resources and Strengthen Management

In order to continuously improve the health status of the elderly, we must make full use of health resources; build a trinity medical service system of hospital, community, and family; and provide continuous and integrated medical and health services for the elderly. In addition, according to the disease needs of the elderly, formulate appropriate nursing plans, and implement relevant measures. While nursing the body of the elderly, we should also strengthen the care of the mental health of the elderly and actively carry out health education for the elderly. Being aware of the physical discomfort can make the elderly face the disease easily and ensure that the existing medical resources can be better utilized and better meet the standard medical treatment of low-income elderly, so as to realize the significance of elderly care services for the elderly.

## 5. Summary

The problem of China's population structure leads to the emergence of the problem of providing for the aged in newborn families. Therefore, it is unrealistic to rely on children to track the old age in the whole process. The nursing service for the elderly has become the focus of today's society. The study took 500 elderly patients in a tertiary hospital in a city as the research object. The survey results show that compared with our medical level, the conditions of nursing institutions are not ideal, the professional ability of nursing staff is low, and the management is not in place, resulting in the dissatisfaction of the elderly, which has seriously affected the quality of life of the elderly in their later years. The vast majority of elderly patients have high requirements for their elderly care services, which is related to family income and other related factors. Therefore, relevant departments should formulate corresponding measures to improve the quality of life of the elderly. Due to the rapid aging of China and the traditional view of raising children and preventing the elderly, the existing social view on the maintenance and management of the elderly is not enough. In the future, this market is huge, and potential business opportunities need to be further developed.

## Figures and Tables

**Figure 1:** The ratio of the researcher and whether care is needed.

**Figure 2:** The ratio of family income and care.

**Figure 3:** The ratio of marital status and care needs of the researcher.

**Figure 4:** The proportion of whether the researchers took care of themselves and needed care.

**Table 1:** General information and service needs of the elderly.

Example number	Degree of education			Marital status		Family income/(yuan/month)			Self-care ability	
500	Junior high school and below	Senior school	College degree or above	Married	Divorce/widowed	<2500	2500~5500	>5500	Can take care of yourself	Cannot take care of yourself
	146	231	123	341	159	112	207	181	374	126
Proportion/%	29.2	46.2	24.6	68.2	31.8	22.4	41.4	36.2	74.8	25.2
Have nursing needs	32	68	102	105	117	21	43	109	51	94
Proportion/%	21.9	29.4	82.9	30.8	73.6	18.8	20.8	60.2	13.6	74.6
P	<0.05									

**Table 2:** Logistics regression analysis of factors of nursing needs.

Equation	Age	Take care of yourself	Education level	Gender	Marital status	Family income
Regression coefficient	0.954	4.013	3.187	0.872	0.963	2.078
Standard error	0.978	1.035	1.096	1.091	1.514	1.801
Wald price	1.054	1.985	1.923	2.564	1.223	1.914
Variance	1	1	1	1	1	1
*P*	0.324	0.509	0.247	0.376	0.208	0.567
95% credibility interval	0.529~18.109	0.517~11.247	0.520~2.948	0.952~20.119	1.024~2.897	0.125~75.295

## Data Availability

The data underlying the results presented in the study are available within the manuscript.
